# Optimal diagnosis of the skin cancer using a hybrid deep neural network and grasshopper optimization algorithm

**DOI:** 10.1515/med-2022-0439

**Published:** 2022-03-11

**Authors:** Gengluo Li, Giorgos Jimenez

**Affiliations:** School of Information Engineering, NanChang University, NanChang, Jiangxi 330031, China; University of Wisconsin-Madison, Madison, WI 53706, USA

**Keywords:** medical imaging, skin cancer, AlexNet, extreme learning machine, improved grasshopper optimization algorithm

## Abstract

When skin cells divide abnormally, it can cause a tumor or abnormal lymph fluid or blood. The masses appear benign and malignant, with the benign being limited to one area and not spreading, but some can spread throughout the body through the body’s lymphatic system. Skin cancer is easier to diagnose than other cancers because its symptoms can be seen with the naked eye. This makes us to provide an artificial intelligence-based methodology to diagnose this cancer with higher accuracy. This article proposes a new non-destructive testing method based on the AlexNet and Extreme Learning Machine network to provide better results of the diagnosis. The method is then optimized based on a new improved version of the Grasshopper optimization algorithm (GOA). Simulation of the proposed method is then compared with some different state-of-the-art methods and the results showed that the proposed method with 98% accuracy and 93% sensitivity has the highest efficiency.

## 1 Introduction

The skin is the protective layer of the body that covers it all around and protects us from sunlight, heat, cold, superficial damage such as wounds and scratches, infection, and penetration of bacteria and viruses. Between the various layers of skin, there are two main layers called the epidermis and dermis that act as a protector. The dermis is a layer that contains blood, hair follicles, and glands. The epidermis contains three main types of cells called squamous cells, basal cells, and melanocytes.

When skin cells divide abnormally, it can cause a tumor or abnormal lymph fluid or blood. The masses appear benign and malignant, with the benign being limited to one area and not spreading, but some can spread throughout the body through the body’s lymphatic system [1]. Skin cancer is easier to diagnose than other cancers because its symptoms can be seen with the naked eye.

The most common causes of skin cancer are exposure to ultraviolet (UV) rays from direct sunlight or exposure to chemicals produced by certain types of light bulbs [2]. These two factors alter the DNA of the cells we talked about above, altering the growth and development of these cells and turning them into cancerous masses [3].

The initial formation of cancer in an organ is called primary cancer. A malignant mass that has not yet spread to other parts of the body is called a local. These masses can grow into their blood vessels by attacking the surrounding tissues. Secondary cancer or metastasis occurs when cancer cells grow elsewhere and form a new mass.

Therefore, the initial diagnosis of skin cancer can be so useful for the early detection of this cancer. Diagnosis of skin cancer is usually possible with a biopsy. But in most cases, this method is a suffering process in both pain and time for the patient. Recently, methods such as dermoscopy have been used to help diagnose suspected lesions, but ultimately a skin biopsy should be used to diagnose the nature of any suspected skin lesions. In recent years, research has been conducted on methods for rapid and accurate diagnosis of skin cancer from dermoscopic images with different diagnostic accuracy. For example, Zhang et al. [4] analyzed the diagnose of skin diseases using an optimum Convolution Neural Network (CNN). Quick diagnose of skin melanoma helps prevent the disease. One of the most widely used methods in the diagnosis of skin diseases is the use of image processing. In this study, a new method of CNN based on the Whale optimization algorithm was used to diagnose melanoma.

Xu et al. [5] diagnosed melanoma diseases using the K-Fuzzy C-, a technique based on the development of the Red fox optimization (RFO) algorithm. In this study, an optimum pipeline process was used to accurately detect the melanoma spots from dermoscopic images. First, after pre-processing of the image, areas of the skin were divided into parts by the C-means Kernel Fuzzy technique. Then, the main features of the divided skin are optimally selected by the optimized algorithm. The results showed that the optimum K-Fuzzy C-means was the accurate diagnosis of melanoma spots on the skin. K-Fuzzy C- a technique based on the development of the RFO algorithm provided more accurate and reliable results in the classification of the skin and the detection of melanoma spots on the skin.

Tan et al. [6] used an intelligent technique to detect melanoma spots on the skin. They used Particle swarm optimization (PSO) methods and deep learning techniques. The deep CNN is optimized by the PSO model. In this research, the PSO method was used to optimize the identification of melanoma areas on the skin. The results of the developed deep CNN were compared with classical methods and statistical tests. The results showed that developed deep CNN had a better ability to detect damaged areas of the skin and melanoma spots compared to classical methods.

Parsian et al. [7] detected melanoma spots in dermoscopic images using the Wildebeest herd optimization (WHO) algorithm. A common method for diagnosing skin cancer is a non-invasive dermatoscopic method based on ocular inference. Therefore, it is difficult for specialists to diagnose melanoma spots on the skin. Therefore, the use of artificial intelligence techniques can increase the accuracy of diagnosing melanoma. In this study, deep learning optimized by WHO algorithm was used to detect melanoma spots on the skin. The suggested model was implemented on the ISIC-2008 skin cancer dataset. The data analysis showed that this method has a high ability to diagnose the disease.

Khamparia et al. [8] used the deep learning method to detect the cancerous spots on the skin. Diagnosis and classification of skin cancer in the early stages of development can increase the possibility of recovery of patients. For this purpose, the CNN was used to distinguish benign from malignant spots. Observation of the results showed good performance of the CNN in the diagnosis and classification of malignant skin lesions.

It can be observed from the literature that there are different research works for the diagnosis of skin cancer from dermoscopy. The results also show that using metaheuristic algorithms for this purpose is exponentially increasing. This study uses a hybrid technique based on deep learning and metaheuristics for the diagnosis of skin cancer. The new metaheuristic is based on an improved version of the Grasshopper optimization algorithm (GOA) which provides results with higher accuracy and precision.

## 2 Materials and methods

### 2.1 Dataset

The designed module is an optimized deep learning-based system that includes a general form to diagnose cancer from the input images, directly. The designed diagnosis in this study has been programmed in MATLAB R2019b environment and its results are verified by applying to a database, called PH^2^ [9]. The PH^2^ database includes some different dermoscopic images that are gathered from the Dermatology Service of Hospital Pedro Hispano (Matosinhos, Portugal) under identical conditions. The dataset includes 8-bit 768 × 560 resolution RGB color images. The total dataset includes 200 dermoscopic images with 80 atypical nevi, 80 common nevi, and 40 melanomas. This database is available at: https://www.fc.up.pt/addi/ph2%20database.html.

The training and the test data for the benchmarks are set at 80 and 20%, respectively. Figure 1 shows some samples in the PH^2^ dataset in this study.

**Figure 1:** Some samples of the PH^2^ dataset in this study.

### 2.2 AlexNet

AlexNet is a family of deep neural networks and a subdivision of the CNN, which is designed by Alex Krizhevsky and Ilya Sutskever, and Geoffrey Hinton [18]. The Alex network does well the diagnosis targets, for example, the classification of the ImageNet dataset with high precision [10]. In this study, we used the batch normalization (BN) technique for improving the AlexNet reliability to be used as a diagnostic system in skin cancer detection. Due to the higher complexity of the database images because of their higher variance in terms of brightness, the distributions of the inputs in AlexNet are different in each layer. This process increases the complexity of the system elapsed time during training of the parameters with good initialization. To resolve this problem, BN has been utilized [11]. With CNN training based on the minibatch technique, a normalization transform is used by the activations of the layer to recall the constant means and variances. So, with a random valuation of a set of variables, ({x}_{i}:i=1,2,\ldots ,n)] , that S] defines their mini-batch values, i.e., S={[}{z}_{1},{z}_{2},\ldots ,{z}_{n}]] , their mean value and variance are formulated as follows:

(1) {\text{mean}}_{\text{S}}=\frac{1}{N}\mathop{\sum }\limits_{j=1}^{N}{z}_{i},]

(2) {\text{StD}}_{\text{S}}^{\text{2}}=\frac{1}{N}\mathop{\sum }\limits_{j=1}^{N}{({z}_{i}-{\text{mean}}_{\text{S}})}^{2}.]

Consequently, the normalized values ( \widehat{{x}_{i}}] ) are modeled as follows:

(3) \widehat{{z}_{i}}=\frac{{z}_{i}-{\text{mean}}_{\text{S}}}{\sqrt{{\text{StD}}_{\text{S}}^{2}+\varepsilon }},]

where *ε* is used for preventing steadiness.

Since, in some cases, the normalized activations are not the purpose of the learning goal, the following transformation is used for that target:

(4) {y}_{i}=a+b\times {\hat{z}}_{i},]

where a] and b] are two adjustable parameters in the minibatch.

By considering the BN, the speed for training in the CNNs has been accelerated, such that their independence increases from the initial values of the parameters. Furthermore, BN adjusts and enhances the networkability generalization.

### 2.3 Extreme learning machine (ELM)

Because of the dependency of the AlexNet to the previous fully connected layers, it is better to improve it to get better results. Therefore, the network is combined with a popular efficient network, called ELM. This report presents the model and its relationship with SVM-based models. These models are in the field of binary classification. Of course, with techniques such as the one against all and one against one, they can be developed in several categories. The ELM is a simplified integration of the PSVM, LS-SVM, and regulatory algorithms. The hidden layers of the ELM model do not need to be tuned, and these layer functions are determined. Therefore, this network has been used for improving the accuracy of the model. A general form of an ELM model has been illustrated in Figure 2.

**Figure 2:** A general form of an ELM model.

In Figure 2, b] defines the bias of the hidden layer, w,] and \beta ] describe the input and output weights, respectively, x] and O] represent the input and output.

An important reason for utilizing the ELM network along with AlexNet for skin cancer diagnosis is that it doesn’t need more iterations for training, which enhances its efficiency in terms of convergence.

With assuming a training set M] :

(5) M={[}({x}_{1},{t}_{1}),({x}_{2},{t}_{2}),\ldots ,({x}_{n},{t}_{n})],]

where {x}_{i}] and {t}_{i}] represent the input vector and label, respectively.

The output matrix for hidden layer H] has been obtained by the following equation:

(6) H=\mathop{\sum }\limits_{l=1}^{N}{f}_{i}\times ({w}_{i}{x}_{i}+{b}_{i}),\hspace{.5em}l=1,2,\ldots ,L,]

where N] describes the number of hidden nodes and f(\cdot )] represents the hidden layer activation function. Finally, the target is to deliver the ELM model output, like the actual sample labels, that is:

(7) H\theta =T,]

where T={[}{t}_{1},{t}_{2},\ldots ,{t}_{L}]] .

So, the \theta ] obtained by the following equation:

(8) \theta ={H}^{t}T,]

where t] defines the pseudo-inverse operator.

As mentioned before, the ELM model has been used to replace the preceding layers to decrease the complexity of the system for the diagnosis purpose.

One important case in designing the weights and biases in the conventional methods is that they are selected randomly. Here to provide a more optimal model for this study, the weights and biases are selected optimally based on a new improved version of the GOA.

## 3 Improved GOA

### 3.1 The concept of GOA

GOA optimization algorithm was presented for the first time in the year 2017 by Hamian et al. [12]. The proposed algorithm is mathematically modeled and proposed inspired by grasshopper attack behavior in nature to solve optimization problems. Grasshoppers are small insects. But because of the damage, they do to agricultural products, they are a serious pest for crops. Although grasshoppers are usually found alone in the wild, they belong to the largest group of insects. The size of a group of grasshoppers can be on a continental scale and can be a big nightmare to the farmers. A unique aspect of grasshoppers is their group behavior in childhood and adulthood. Millions of baby grasshoppers jump and move like rolling hoses, eating and destroying almost every product in their path.

When they grow up, they form groups in the air and travel long distances to migrate. The main feature of the grasshopper group in the larval stage is their slow movement and small steps. In contrast, sudden movement is the main feature of larger grasshoppers. Searching for food is another important feature of the grasshopper group.

The main article of the GOA claims that grasshopper life inherently has both exploitation and exploration. In this way, immature grasshoppers have smooth and continuous movements, and next to them, adult grasshoppers have completely random and mutant movements. Therefore, they have the role of exploitation and exploration, respectively. As a result, modeling the GOA leads to the creation of a powerful and appropriate algorithm [13].

Therefore, if this behavior is mathematically modeled, a new nature-inspired algorithm can be designed. The mathematical model used to simulate the group behavior of grasshoppers is as follows:

(9) {X}_{i}={S}_{i}+{G}_{i}+{A}_{i},]

where {X}_{i}] is the position of the i] grasshopper, {S}_{i\text{ }}] is the social interaction, {G}_{i}\text{ }] is the gravitational force in the i] grasshopper, and {A}_{i\text{ }}] is the horizontal motion of the wind. Note that to create a random behavior, the equation can be written as {X}_{i}={r}_{1}{S}_{i}+{r}_{2}{G}_{i}+{r}_{3}{A}_{i}] where {r}_{1,}\text{ }{r}_{2}] , and {r}_{3}] are random numbers in the range {[}0,\text{ }1]] . The {S}_{i}\text{ }] function, which defines social interaction, is calculated as follows:

(10) {S}_{i}=\mathop{\sum }\limits_{j}^{N}=s({d}_{ij}){\hat{d}}_{ij},\hspace{.5em}j\ne i,]

where {d}_{ij\text{ }}] is the distance between grasshopper i] and grasshopper j] and is calculated as {d}_{ij}=| {X}_{j}-{X}_{i}| ] , S] is a function to define the power of social forces, and {\grave{d}}_{ij}=\frac{{X}_{j}-{X}_{i}}{{d}_{ij}}] is a single vector of grasshopper i] to the grasshopper j] . The function S] , which defines social forces, is calculated as follows:

(11) S(r)=f{\text{e}}^{\frac{-r}{l}}-{\text{e}}^{-r},]

where f] represents the adsorption intensity and l] represents the adsorption length scale. The {G}_{i}\text{ }] factor in Equation is calculated as follows:

(12) {G}_{i}=-g\cdot {\bar{e}}_{\text{g}},]

where g] is the constant of gravity and {e}_{\text{g}}] represents a single vector toward the center of the earth. The factor {A}_{i\text{ }}] in equation is calculated as follows:

(13) {A}_{i}=u\cdot {\bar{e}}_{\text{w}},]

where u] is a floating object constant and *e*_w_ is a unit vector in the wind direction. Baby grasshoppers have no wings. As a result, their motion is highly dependent on the wind direction. By substituting G] , S,] and A] in Equation this equation can be defined as follows:

(14) {X}_{i}=\mathop{\sum }\limits_{j=1,i\ne j}^{N}s(| {X}_{j}-{X}_{i}| )\frac{{X}_{j}-{X}_{i}}{{d}_{ij}}-g\times {\bar{e}}_{\text{g}}+u\times {\bar{e}}_{\text{w}}.]

The situation update is as follows:

(15) {X}_{i}=\beta \times \left(\mathop{\sum }\limits_{j=1,i\ne j}^{N}\beta \times \frac{u{b}_{d}-l{b}_{d}}{2}\times s\times (| {x}_{j}^{d}-{x}_{i}^{d}| )\times \frac{{x}_{j}-{x}_{i}}{{d}_{ij}}\right)+{\bar{T}}_{d},]

where \text{ }u{b}_{d\text{ }}] is the upper range in the D] dimension, l{b}_{d}] is the low range in the D] dimension, d] is the value of the D] dimension in the target (the best solution obtained), and \beta \text{ }] is the reduction coefficient to minimize the neutral zone and the gravity-repulsion zone.

The equation shows that the next position of a grasshopper is defined based on the current position, the target position, and the position of the other grasshoppers. Note that the first factor in this equation is the current position of the grasshopper relative to the other grasshoppers. Keep in mind that all grasshoppers need to be able to determine the position of the search agents around the target.

To balance exploration and exploitation, a parameter is needed to reduce repetition. This increases the utilization factor, while also increasing the repetition rate. Parameter \beta \text{ }] has been used twice in the above equation for the following reasons:

- Intra-sigma coefficient \beta \text{ }] reduces the gravitational-repulsive zone and the neutral zone between the grasshoppers.
- The coefficient \beta \text{ }] outside Sigma strikes a balance between exploration and exploitation

To balance the two characteristics of exploration and operation, the update coefficient is considered as a geometric sequence, which is calculated as follows:

(16) \beta ={\beta }_{\text{max}}-{\left(\frac{\text{It}}{\text{MaxIt}}\right)}^{w}({\beta }_{\text{max}}-{\beta }_{\text{min}}),]

where {\beta }_{\text{max}}] is the maximum value and {\beta }_{\text{min}}] is the minimum value, w] is the geometric coefficient, it is the current iteration, and \text{MaxIt}] is the maximum number of iterations. For this purpose, the update coefficient w is calculated as follows:

(17) W={W}_{\text{max}}-it\frac{{W}_{\text{max}}-{W}_{\text{min}}}{\text{MaxIt}},]

where {W}_{\text{max}}] is the maximum and {W}_{\text{min}}] is the minimum, it is the current iteration, and \text{MaxIt}] is the maximum iteration.

### 3.2 Improved GOA

The original GOA has some shortcomings like premature convergence and lower consistency. This issue motivates us to design an improved version of this algorithm with modifications on it about the aforementioned issues. Here we used two modifications to improve the algorithm.

#### 3.2.1 The quasi-oppositional learning (quasi-OBL)

Quasi-oppositional learning is studied here to improve the convergence speed of the algorithm. Based on the OBL mechanism, the randomly generated candidate has been compared with its symmetric value to select the best one during the process [14].

By considering the i\text{th}] integer ({X}_{i})] in a *D*-dimensional search space with \text{Lb}] and \text{Ub}] as lower and upper limitations, the symmetric value has been obtained by the following equation:

(18) {\bar{X}}_{i}={\text{Lb}}_{i}+{\text{Ub}}_{i}-{X}_{i},]

where, i=1,2,\ldots ,D] .

Besides, the quasi-opposite value ({\breve{X}}_{i})] of the i\text{th}] integer ( {X}_{i}] ) is obtained by the following equation:

(19) {\breve{X}}_{i}=r\hspace{.25em}\text{and}\hspace{.25em}({X}_{i},\hspace{.25em}0.5\times {\text{Lb}}_{i}+{\text{Ub}}_{i}).]

#### 3.2.2 Merit function (MF)

The MF is another modification that can be utilized for improving the algorithm consistency. This mechanism provides a proper balance between exploration and exploitation. Based on this mechanism, the optimization process begins with large steps (exploration), and then, it gradually decreases its steps (exploitation). The MF can be formulated as follows:

(20) X(t+1)=\left\{\begin{array}{c}\frac{mF({X}_{i-1})}{mF({X}_{i-1})}X(t),\hspace{.25em}mF({X}_{i})\ge mF({X}_{i-1})\\ {X}_{i},\hspace{.25em}mF({X}_{i})\lt mF({X}_{i-1}),\end{array}\right.]

where mF({X}_{i})] describes the MF that is obtained as follows:

(21) mF({X}_{i})={X}_{i}-\frac{{\nabla }^{T}g({X}_{i})X(t)}{{\nabla }^{T}g({X}_{i})\nabla g({X}_{i})}\nabla g{(X(t))}^{2}+\frac{{({X}_{i})}^{2}}{{({X}_{0})}^{2}},]

where {X}_{0}] and {\nabla }^{T}g({\text{X}}_{i})] signify random value and the gradient vector of g({X}_{i}^{j})] at point {X}_{i}] .

### 3.3 Algorithm authentication

To validate the effectiveness of the proposed improved GOA, it has been applied to four standard benchmark functions including two unimodal and two multimodal basic functions including Schwefel 2.22 function, Sphere function, Quartic function, and Rosenbrock function. The studied functions are explained completely in the following.

*Schwefel 2.22*: a function with 30 dimensions that is limited in the range [−10, 10]. The formula for this function is as follows:

(22) {F}_{1}(x)=\mathop{\sum }\limits_{i=1}^{n}|{X}_{i}|+\mathop{\prod }\limits_{i=1}^{n}|{x}_{i}|.]

*Sphere*: a function with 30 dimensions that is limited in the range [−100, 100]. The mathematical formula for this function is as follows:

(23) {F}_{2}(x)=\mathop{\sum }\limits_{i=1}^{n}{x}_{i}^{2}.]

*Quartic:* a function with 30 dimensions that is limited in the range [−128, 128]. The mathematical formula for this function is as follows:

(24) {F}_{3}(x)=\mathop{\sum }\limits_{i=1}^{n}i{x}_{i}^{4}+\text{random}{[}0,1)\text{ }\text{.}]

*Rosenbrock:* a function with 30 dimensions that is limited in the range [−30, 30]. The mathematical formula for this function is as follows:

(25) {F}_{4}(x)=\mathop{\sum }\limits_{i=1}^{n-1}{[}100{({x}_{i+1}-{x}_{i}^{2})}^{2}+{({x}_{i}-1)}^{2}],]

where the minimum value of all the abovementioned functions is 0.

To verify the efficiency of the proposed improved GOA, it is compared with some popular and new algorithms including Black hole (BH) [15], Multi-verse optimizer (MVO) [16], Emperor penguin optimizer (EPO) [17], and the original GOA [18].

– BH [15]:

a={[}0,1]] ; number of stars = 100
– MVO [16]:
  Traveling distance rate = [0.6, 1]; Wormhole existence prob. = [0.2, 1]
– EPO [17]

\overrightarrow{A}=1] ; {T}^{^{\prime} }=100] ; M=2] ; f=2] ; S=1] ; l=1.5] .
– Bat Optimization [19]

\alpha =0.9] ; \gamma =0.9] .
– GOA [12]

{c}_{\text{min}}=1] ; {c}_{\text{max}}=0.00001] .

Due to the stochastic behavior of the presented improved GOA, it is run 30 times, independently.

To get a fair analysis, the maximum iteration number is set at 200 and the population size is set at 35. The programming has been implemented on a 64-bit MATLAB R2019b environment. The configuration of the system is given in Table 1.

**Table 1:** The configuration of the system

Name	Setting
Hardware	Intel^®^ Core™ i7-4720HQ
CPU	1.60 GHz
RAM	16 GB
Frequency	1.99 GHz
Operating system	Windows 10
Programming software	MATLAB R2019b

Table 2 indicates the simulation results of the presented improved GOA and its comparison with some state-of-the-art metaheuristics based on the mean value (MEAN) and the standard deviation (SD) value.

**Table 2:** The simulation results of the suggested improved GOA compared with other studied algorithms

Algorithm		Sphere	Schwefel 2.22	Quartic	Rosenbrock
BH [15]	Min	6.5483	0.0125	0.0098	8.2547
	Max	3.2648 × 10^2^	2.2648 × 10^2^	1.3471 × 10^3^	0.2871 × 10^4^
	AVE	2.2543 × 10^2^	2.0147 × 10^2^	2.8471 × 10^3^	25.3487
	SD	2.0582 × 10^4^	1.9347 × 10^2^	2.0841 × 10^3^	20.3481
MVO [16]	Min	5.0348	1.0095	1.0041	2.4275
	Max	254.3547	25.3147	9.1079	32.1284
	AVE	145.2648	11.2647	5.2217	25.2647
	SD	98.3547	10.2648	4.9647	14.2517
EPO [17]	Min	3.9824	5.3473 × 10^−3^	2.859 × 10^−3^	1.2174
	Max	201.6484	9.6471	5.0054	2.0364
	AVE	82.2648	7.0021	2.0417	0.8217
	SD	75.2648	5.0647	1.1654	0.6314
GOA [18]	Min	1.2543	1.3481 × 10^−5^	1.2517 × 10^−6^	2.2581 × 10^−7^
	Max	95.3487	1.6471 × 10^−4^	4.2476 × 10^−5^	0.6174 × 10^−6^
	AVE	6.2648	1.1048 × 10^−4^	3.1507 × 10^−5^	1.6174 × 10^−6^
	SD	44.2648	0.9421 × 10^−4^	4.5973 × 10^−5^	1.3416 × 10^−6^
IGOA	Min	0.9358	6.3247 × 10^−9^	5.0641 × 10^−10^	3.5176 × 10^−12^
	Max	55.0254	1.6471 × 10^−8^	1.9437 × 10^−9^	0.3728 × 10^−11^
	AVE	2.3647	1.2517 × 10^−8^	2.6351 × 10^−9^	1.3481 × 10^−11^
	SD	1.0254	1.1638 × 10^−8^	2.1647 × 10^−9^	1.0581 × 10^−11^

As can be inferred from Table 2, the presented IGOA has the minimum value of the results in terms of the mean value for all four benchmark functions which indicates the better accuracy of this algorithm toward the comparative algorithms. Also, on checking the standard deviation in the proposed algorithm, the minimum value of this parameter in the functions shows its higher consistency toward the other state-of-the-art algorithms.

## 4 The proposed network

This part of the article explains the method of optimization for the proposed combined AlexNet and ELM net by considering the batch normalized technique and the design improved GOA. The method starts with a pre-trained AlexNet for extracting the features from the dermoscopy images. To resolve the internal covariate shifting problem, BN is performed on the layers. Because of the number of classes in this study, i.e., cancerous and normal, the last three layers of the pre-trained network should be modified. Because the default output number for this network is 1,000 nodes.

We also added six numbers of normalization layers, after the convolution and pooling layers. Finally, the ELM network has been addended as the classifier part of the AlexNet. The best numbers of the layers are achieved based on trials and errors. For optimal designing of the ELM model, its weights and biases are optimally selected based on the proposed improved GOA. To use the proposed IGOA for the network optimization, the following objective function has been utilized:

(26) f(w,b)=\mathop{\displaystyle \sum }\limits_{j=1}^{N}{({d}_{j}-{y}_{j})}^{2},]

where N] defines the number of training samples, d] and {y}_{i}] describe the output of the ELM network and the image label, respectively.

## 5 Experimental results

The performance analysis has been evaluated based on six parameters, accuracy, specificity, precision, *F*1 score, sensitivity, and Matthew’s correlation coefficient (MCC). The mathematical model of the mentioned measure formulations has been given below:

(27) \text{Specificity}=\frac{\text{TN}}{\text{TN}+\text{FP}}\times 100,]

(28) \text{Accuracy}=\frac{\text{TP}+\text{TN}}{\text{TP}+\text{TN}+\text{FP}+\text{FN}}\times 100,]

(29) \text{Precision}=\frac{\text{TP}}{\text{TP}+\text{FP}}\times 100,]

(30) \text{Sensitivity}=\frac{\text{TP}}{\text{TP}+\text{FN}}\times 100,]

(31) F1\text{-score}=2\times \frac{\text{Precision}\times \text{Sensitivity}}{\text{Precision}+\text{Sensitivity}}\times 100,]

(32) \text{MCC}=\frac{\text{TP}\times \text{TN}-\text{TP}\times \text{FN}}{\sqrt{(\text{TP}+\text{FP})\times (\text{TP}+\text{FN})\times (\text{TN}+\text{FP})\times (\text{TN}+\text{FN})}}\times 100,]

where TP, TN, FP, and FN represent the true positive, true negative, false positive, and false negative, respectively.

Table 3 illustrates the performance analysis of the proposed method toward some other state-of-the-art methods including AlexNet [20], CNN [21], and RCNN [22] (Figure 3).

**Table 3:** The performance analysis of the proposed method toward some other state of the art methods

Method	Accuracy	Precision	Specificity	*F*1-score	Sensitivity	MCC
AlexNet [20]	0.85	0.95	0.97	0.86	0.77	0.56
CNN [21]	0.97	0.94	0.95	0.95	0.94	0.91
RCNN [22]	0.90	0.91	0.94	0.95	0.90	0.88
AlexNet-ELM-IGOA	0.98	0.96	0.98	0.94	0.93	0.91

**Figure 3:** The classification analysis of the proposed method toward some other state of the art methods.

From Table 3, it has been experimentally proved that the proposed AlexNet-ELM-IGOA technique outperforms the other analyzed methods. For more clarification, it is clear that the proposed methodology with 98% accuracy, 96% precision, 96% specificity, 94% *F*1-score, 93% sensitivity, and 91% MCC has the highest values for all the measurements.

To provide more analysis for the proposed AlexNet-ELM-IGOA technique, its results are compared with some other methods including Brinker et al. [23], Mustafa and Kimura [24], Babino et al. [25], Hagerty et al. [26], and Bi et al. [27] from literature. To perform the analysis, sensitivity, accuracy, specificity, and negative predictive value (NPV), and positive predictive value (PPV) measures are utilized where:

(33) \text{PPV}=\frac{\text{TP}}{\text{TP}+\text{FP}}\times 100,]

(34) \text{NPV}=\frac{\text{TN}}{\text{TN}+\text{FN}}\times 100,]

The comparison results of the simulation are given in Table 4.

**Table 4:** The comparison results of the simulation

Method	Sensitivity	Specificity	PPV	NPV	Accuracy
Proposed Method	0.93	0.98	0.86	0.88	0.98
Brinker et al. [23]	0.84	0.86	0.78	0.81	0.84
Bi et al. [27]	0.79	0.75	0.68	0.87	0.75
Hagerty et al. [26]	0.75	0.72	0.64	0.83	0.72
Mustafa and Kimura [24]	0.74	0.72	0.63	0.85	0.70
Babino et al. [25]	0.80	0.88	0.79	0.76	0.82

To provide a graphical clarification, the results are also shown in Figure 4.

**Figure 4:** The classification analysis of the proposed method toward some other state of the art methods.

As can be seen from Table 3 and Figure 4, the proposed method has the highest accuracy again which shows its superiority toward the second series comparative algorithms; however, Brinker et al. and Babino et al. methods with 84 and 82% are placed in the second and the third ranks. Then, Bi’s method with 75% accuracy, Hagerty’s method with 72%, and Mustafa’s with 70% accuracy are in the next positions. Likewise, the proposed method with 93% sensitivity provides the highest reliability in solving the diagnosis problem. A higher value of the specificity (98%) of the proposed method toward the others specifies its sophisticated occurrence-independent values.

## 6 Conclusion

Melanoma is the most dangerous skin cancer with a high mortality rate, and the most worrying thing is that the more fashionable tanning becomes in the world, the higher the incidence of this disease. The main benefit of diagnosing the first symptoms of melanoma is seeing a doctor and getting treatment very quickly, which will be more helpful. One non-destructive test for this purpose is to use dermoscopy images. To reduce human errors, recently, image processing and artificial intelligence techniques have been utilized. Therefore, in this study, a new configuration of the deep learning based on the AlexNet and ELM network was utilized to provide better results of the diagnosis. To get better results, the weights and biases of the network were optimally selected based on an improved version of the GOA. The final results showed that the proposed method with 98% accuracy and 93% sensitivity provides the highest accuracy compared to the other methods.
